# Perinatal Outcomes and Related Risk Factors of Single vs Twin Pregnancy Complicated by Gestational Diabetes Mellitus: Meta-Analysis

**DOI:** 10.1155/2022/3557890

**Published:** 2022-07-04

**Authors:** Xiaofang Zhu, Chan Huang, Li Wu, Yufeng Deng, Xuemei Lai, Huayan Gu, Haiyan Zhang

**Affiliations:** Department of Obstetrics and Gynecology, Women and Children's Hospital of Chongqing Medical University, Chongqing 401147, China

## Abstract

**Objective:**

Perinatal outcomes and related risk factors of single vs twin pregnancy complicated with gestational diabetes mellitus (GDM) were clarified, providing evidence for developing preventive measures.

**Methods:**

The Chinese National Knowledge Infrastructure (CNKI), China Biology Medicine (CBM), CQVIP, Wanfang, and PubMed databases were searched for published research on the perinatal outcomes and risk factors of single and twin pregnancy complicated by GDM from 2000 to 2021. The quality of the included literature was evaluated according to the Newcastle-Ottawa Scale (NOS). Meta-analysis of the included literature was conducted using RevMan5.3 software.

**Results:**

Relative to a single pregnancy group, infertility, gestational weight gain, and family history of diabetes presented statistical significance in the twin pregnancy group (*P* < 0.05); gestational age at delivery, cesarean section, preterm birth < 37 weeks, and preeclampsia presented statistical significance in the twin pregnancy group (*P* < 0.05); and neonatal birth weight, small for gestational age (SGA), neonatal asphyxia, neonatal hypoglycemia, neonatal respiratory distress syndrome (NRDS), neonatal hyperbilirubinemia, and neonatal death presented statistical significance in the twin pregnancy group (*P* < 0.05).

**Conclusion:**

Infertility, prenatal weight gain, and diabetes in the family are all risk factors for postpartum impaired glucose metabolism in pregnant women with GDM who are carrying twins. The gestational age at delivery, cesarean section, preterm birth < 37 weeks, and preeclampsia of twin pregnant women with diabetes will affect the perinatal status of twin pregnant women. Neonatal birth weight, SGA, neonatal asphyxia, neonatal hypoglycemia, NRDS, neonatal hyperbilirubinemia, neonatal death, etc. should be paid special attention in the perinatal process.

## 1. Introduction

Gestational diabetes mellitus (GDM) is the most common metabolic disease in pregnancy, and its incidence is increasing globally due to elevated obesity in women of childbearing age, elderly parturient women, and assisted reproductive technologies. Incidence of GDM in twin pregnancy presents elevation relative to single pregnancy, and twin pregnancy is an independent risk factor for GDM occurrence [1, 2].

Preterm birth, infection, macrosomia, polyhydramnios, postpartum hemorrhage, newborn hypoglycemia, neonatal respiratory distress syndrome (NRDS), neonatal hypercholesterolemia, and other perinatal problems have all been linked to GDM in single pregnancies [3]. There are different opinions at home and abroad about whether GDM will increase the adverse pregnancy outcome of twin pregnancy. The related risk factors and early prediction research of GDM also focus on single pregnancy, and reports on twin pregnancy are rare. Understanding the perinatal outcomes and risk factors of GDM, as well as GDM prevention, early diagnosis, and early treatment, is critical for enhancing the quality of life of pregnant and lying-in women, as well as perinatal infants.

The following is the paper's organization paragraph: in Section 2, the materials and methods is provided. The experiments and results are discussed in Section 3.  Section 4 consists of the discussion; finally, the research job is completed in Section 5.

## 2. Materials and Methods

In this section, we defined the data source, literature inclusion criteria, literature exclusion criteria, literature screening and data extraction, quality evaluation, and statistical analysis in detail.

### 2.1. Data Source

The China National Knowledge Infrastructure (CNKI), China Biology Medicine (CBM), CQVIP, Wanfang, and PubMed databases were retrieved, combined with literature tracing and manual retrieval using the combination of subject headings and keywords. The literatures published on the risk factors of GDM in Chinese women from January 2000 to December 2021 were collected. The literature retrieval terms were as follows: “single vs twin pregnancies,” “gestational diabetes mellitus,” “risk factors,” “perinatal outcomes,” and “case-control study.”

### 2.2. Literature Inclusion Criteria

1. A case-control study
2. Clinically confirmed GDM cases in a case group
3. OR value and its 95% CI being provided or possibly being obtained indirectly by calculation
4. For the report of the same population, a recently published literature being chosen

### 2.3. Literature Exclusion Criteria

1. The study did not set up a control group
2. The diagnostic criteria for GDM were not mentioned or were not clear
3. The unavailable literatures were published repeatedly, with poor quality and incomplete data

### 2.4. Literature Screening and Data Extraction

Two researchers screened the literature and extracted data according to the inclusion and exclusion criteria, respectively, and crosschecked to exclude bias. If there was any disagreement, two researchers discussed it first and negotiated with a third party to resolve it if necessary. The literature data were extracted using Excel, including key elements of literature quality evaluation (title, author, publication time, and sample size), exposure factors (included when there were ≥ 3 literature reports), and outcome measurement data.

### 2.5. Quality Evaluation

Two researchers evaluated the quality of the included literature according to the Newcastle-Ottawa Scale (NOS), which included 3 dimensions and 8 items in total, with a full score of 9 points. A total score of ≤4 was considered low quality, 5–6 was considered moderate quality, and ≥7 was considered high quality. If there was a disagreement in the evaluation results, two researchers discussed it first and negotiated with a third party to resolve it if necessary.

### 2.6. Statistical Analysis

Meta-analysis was conducted using RevMan5.3 software. Results were expressed as odds ratio (OR) with 95% confidence intervals (95% CI). The *χ*^2^ test evaluated the heterogeneity of the included literature (the test level was *α* = 0.05), and the size of the heterogeneity was evaluated according to the *I*^2^ value. When *P* > 0.05 and *I*^2^ ≤ 50%, it indicated that the heterogeneity of the results in each study presented no statistical significance and a fixed-effects model (FEM) was used for meta-analysis; when *P* ≤ 0.05 and *I*^2^ > 50%, it indicated that the study results presented statistical significance; a random-effects model (REM) was used for meta-analysis after excluding clinical heterogeneity. Sensitivity analysis determined whether the combined results of exposure factors were stable.

## 3. Results

### 3.1. Literature Screening Process and Results

EndNote X9 was utilized to reduplicate a total of 1725 linked literatures found through retrieval. After preliminary screening by reading the title and abstract and rescreening by reading the full text, 11 studies were finally included, with a total of 383752 subjects, including 376563 cases in the single pregnancy group (control group) and 7189 cases in the twin pregnancy group (experimental group) (Figure 1).

### 3.2. General Characteristics and Quality Evaluation of Included Literature

A total of 11 case-control reports were included in this study, and the NOS score was 5 for 1 literature, 6 for 5 literatures, 7 for 3 literatures, and 8 for only 2 literatures (Table 1).

### 3.3. Meta-Analysis Results

#### 3.3.1. Analysis of Related Risk Factors

Family history of diabetes and pre-BMI presented no difference in the heterogeneity test (*P* > 0.1 or *I*^2^ < 50%), and FEM was used for analysis; other risk factors presented statistical significance in the heterogeneity test (*P* ≤ 0.1 or *I*^2^ > 50%), and REM was used for analysis. Relative to the single pregnancy group, infertility, gestational weight gain, and family history of diabetes presented statistical significance in the twin pregnancy group (*P* < 0.05), indicating that infertility, gestational weight gain, and family history of diabetes are risk factors for twin pregnant women with GDM. Age and pre-BMI presented no difference after combination (Table 2).

#### 3.3.2. Analysis of Perinatal Outcomes of Pregnant Women

Perinatal outcome indicators of gestational age at delivery, cesarean section, preterm birth < 37 weeks, gestational hypertension, and preeclampsia presented statistical significance in the heterogeneity test (*P* ≤ 0.1 or *I*^2^ > 50%), and REM was used for analysis. Relative to the single pregnancy group, gestational age at delivery, cesarean section, preterm birth < 37 weeks, and preeclampsia presented statistical significance (*P* < 0.05), indicating that gestational age at delivery, cesarean section, preterm birth < 37 weeks, preeclampsia, and gestational diabetes mellitus are important indicators of perinatal outcomes in twin pregnant women with GDM. Gestational hypertension presented no difference after combination (Table 3).

#### 3.3.3. Analysis of Perinatal Outcomes of Neonates

Perinatal outcome indicators of neonatal SAG, neonatal hypoglycemia, neonatal hyperbilirubinemia, and neonatal death presented no difference in the heterogeneity test (*P* > 0.1 or *I*^2^ < 50%); FEM was used for analysis; neonatal birth weight, large for gestational age (LGA), neonatal asphyxia, and NRDS (*P* ≤ 0.1 or *I*^2^ > 50%) presented statistical significance in the heterogeneity test; REM was used for analysis. Relative to the single pregnancy group, neonatal birth weight, SGA, neonatal asphyxia, neonatal hypoglycemia, NDS, neonatal hyperbilirubinemia, and neonatal death presented statistical significance (*P* < 0.05). LGA presented no difference after combination (Table 4).

#### 3.3.4. Analysis of Publication Bias

The funnel plots were essentially symmetrical, according to the literature included in the meta-analysis (Figure 2), suggesting that the meta-analysis results are less likely to have publication bias.

## 4. Discussion

### 4.1. Analysis of Risk Factors for GDM in Twin Pregnancy

At present, domestic and foreign studies generally believe that GDM may be the result of the combined effect of genetic factors and social environmental factors. Though academics at home and abroad have done a lot of research on the risk factors for GDM and have achieved a lot of new discoveries and understandings, earlier publications' results aren't always consistent [15]. Currently identified risk factors are race, advanced pregnancy, prolificacy, family history of diabetes, obstetric history, and overweight. Herein, meta-analysis systematically evaluated the risk factors of GDM by synthesizing the epidemiological research results on the risk factors of GDM in Chinese women in the past 21 years. The study analyzed 11 Chinese and English literatures, and the results demonstrated that infertility, gestational weight gain, and family history of diabetes were the risk factors for postpartum abnormal glucose metabolism in twin pregnant women complicated with GDM. According to one study, prepregnancy overweight or obesity is an independent risk factor for GDM [16], which could be linked to obese people's increased insulin resistance and decreased glucose tolerance. Controlling prepregnancy obesity is a critical step in preventing GDM. Young et al. have revealed that among those with abnormal OGTT during pregnancy, the risk of postpartum diabetes in obese prepregnancy was 22.4 times that of normal weight [17]. Thus, pregnant women with a family history of diabetes should have a reasonable diet and controlling prepregnancy obesity and gestational weight gain is a crucial measure to prevent GDM occurrence. Pregnant women with propregnancy obesity should be more monitored, prenatal examinations should be carried out on time, and GDM should be detected and diagnosed early, so as to reduce the risk of maternal and infant complications.

Analysis of perinatal outcomes in twin pregnancies with GDM: twin pregnancy has been linked to a higher risk of caesarean delivery, GDM, preeclampsia, and preterm birth, but the extent to which GDM enhances the maternal and fetal risk associated with twin pregnancy is unknown. At present, there is no unified conclusion in domestic and foreign studies. Xiao et al. retrospectively analyzed 197 twin pregnancies and believed that GDM did not increase the adverse perinatal outcome of twin pregnancy [18]; Li et al. retrospectively analyzed the clinical data of 329 dichorionic twin pregnancies and concluded that GDM did not increase the adverse perinatal outcomes of dichorionic twin pregnancy [19]. Australian scholars Ooi and Wong retrospectively analyzed the perinatal outcomes of 410 twin pregnancies, of which 99 were diagnosed with GDM, and discovered that twin pregnancies with GDM were more prone to the occurrence of preterm birth, gestational hypertension, and preeclampsia. The incidence of neonatal intensive care unit (NICU) admission and perinatal mortality presented elevation, concluding that twin pregnancies with GDM are a high-risk group with a high incidence of adverse pregnancy outcomes [20]. The meta-analysis of McGrath et al. in 2017 concluded that gestational age and incidence of LGA and SGA presented no difference between GDM twins and non-GDM twins. Twins with GDM has no association with RDS, hypoglycemia, and 5 min Apgar score < 7 points, whereas twin neonates with GDM had a higher chance of being admitted to NICU [21]. Australian scholars Sheehan et al. studied 194 twin pregnancies, of which 39 were complicated with GDM, and believed that in addition to neonatal hypoglycemia, GDM did not increase other adverse perinatal outcomes of twin pregnancy [22]. Hiersch et al. conducted a retrospective cohort study analysis [23]. The research subjects included twin and single live births in Canada from 2012 to 2016. A total of 270843 cases were included, including 266942 single cases, among which 16731 cases were complicated with GDM, with single GDM incidence of 6.3%, and 3901 twin cases, among which 326 cases were complicated with GDM, with twin GDM incidence of 8.3%. No matter in single or twin pregnancy, GDM was related to cesarean section delivery, preterm birth < 37 weeks, and preterm birth < 34 weeks. GDM can raise the risk of gestational hypertension and preeclampsia in a single pregnancy, but not in a twin pregnancy. In terms of neonatal pregnancy outcomes, the rates of neonatal NICU hospitalization, RDS, and hypoglycemia were higher in single GDM but not in twin GDM and the incidence of LGA and neonatal jaundice was higher in single GDM but not in twin GDM. Collectively, relative to single pregnancy, twin GDM has no association with hypertensive disorders complicated with pregnancy and certain neonatal diseases. Nonetheless, the research still highlighted that GDM has association with several adverse pregnancy outcomes in twin pregnancy, including increased cesarean delivery and preterm birth rates and impaired twin fetal growth and development. Herein, relative to the single pregnancy group, five perinatal outcome indicators of gestational age at delivery, cesarean section, preterm birth < 37 weeks, and preeclampsia presented statistical significance in the twin pregnancy group (*P* < 0.05). The analysis of neonatal perinatal outcomes demonstrated that, relative to single pregnancy group, eight perinatal outcome indicators of neonatal birth weight, SGA, neonatal asphyxia, neonatal hypoglycemia, NRDS, neonatal hyperbilirubinemia, and neonatal death presented statistical significance in the twin pregnancy group (*P* < 0.05), suggesting that neonatal birth weight, SGA, neonatal asphyxia, neonatal hypoglycemia, NRDS, neonatal hyperbilirubinemia, and neonatal death are vital indicators for neonatal perinatal outcomes of twin pregnancy complicated by diabetes. LGA presented no difference after combination.

The results of this research are also limited by multiple factors:

1. The number of included literatures is small, and the sample content of each literature varies greatly
2. GDM screening methods and diagnostic criteria used in different literatures are different. However, due to the small number of included literatures, this study did not conduct a stratified analysis of risk factors generated from various diagnostic criteria, which may have influenced the accuracy of the results
3. Meta-analysis itself is a secondary analysis, and there is publication bias, positioning bias, citation bias, etc. The authenticity and validity of its analysis results also largely depend on the quality of original literatures

## 5. Conclusion

In conclusion, infertility, gestational weight gain, and family history of diabetes are risk factors for postpartum abnormal glucose metabolism in twin pregnant women with GDM and these factors are both independent and mutually influencing. To avoid and limit the occurrence and development of postpartum abnormal glucose metabolism in pregnant women with GDM, clinical medical staff should focus on the prevention and regulation of these factors. Moreover, gestational age at delivery, cesarean section, preterm birth < 37 weeks, and preeclampsia of twin pregnant women complicated by diabetes will affect the perinatal status of twin pregnant women. Neonatal birth weight, SGA, neonatal asphyxia, neonatal hypoglycemia, NRDS, neonatal hyperbilirubinemia, neonatal death, etc. should be paid special attention in the perinatal process.

## Figures and Tables

**Figure 1:** Flowchart of literature screening.

**Figure 2:** Funnel plots.

**Table 1:** Literature quality evaluation.

Author	Year	Groups		NOS score
		Single pregnancy group	Twin pregnancy group	
Buhling et al., [4]	2003	178	89	6
Jung et al., [5]	2015	3435	143	6
Lai et al., [6]	2012	327198	5552	5
Rauh-Hain et al., [7]	2009	22503	553	7
Akiba et al., [8]	2019	451	20	8
Morikawa et al., [9]	2015	3667	110	6
Ashwal et al., [10]	2021	1893	180	7
González González et al., [11]	2014	39	39	6
Guillén-Sacoto et al., [12]	2018	240	120	7
Hiersch et al., [13]	2018	16,731	326	8
Weiner et al., [14]	2018	228	57	6

**Table 2:** The related risk factors.

Exposure factors	Number of literatures	Heterogeneity test			OR (95% CI)	*P*
		*I* ^2^ (%)	*P*	Effect model		
Age	10	93	<0.00001	REM	0.46 [−0.42, 1.33]	0.31
Infertility	8	95	<0.00001	REM	1.94 [1.03, 3.67]	0.04
Gestational weight gain	4	96	<0.00001	REM	3.80 [1.08, 6.52]	0.006
Family history of diabetes	5	52	0.08	FEM	1.31 [1.19, 1.44]	<0.00001
Pre-BMI	9	20	0.26	FEM	−0.09 [−0.30, 0.11]	0.37

**Table 3:** Perinatal outcomes of pregnant women.

Perinatal outcome indicators	Number of literatures	Heterogeneity test			OR (95% CI)	*P*
		*I* ^2^ (%)	*P*	Effect model		
Gestational age at delivery	6	98	<0.00001	REM	−3.37 [−3.77, −2.97]	<0.00001
Cesarean section	5	99	<0.00001	REM	4.79 [1.68, 13.67]	0.003
Preterm birth < 37 weeks	5	92	<0.00001	REM	13.47 [5.67, 32.02]	<0.00001
Gestational hypertension	5	71	0.008	REM	0.98 [0.27, 3.53]	0.98
Preeclampsia	3	72	0.03	REM	2.46 [1.48, 4.08]	0.0005

**Table 4:** Perinatal outcomes of neonates.

Perinatal outcome indicators	Number of literatures	Heterogeneity test			OR (95% CI)	*P*
		*I* ^2^ (%)	*P*	Effect model		
Neonatal birth weight	4	61	0.050	REM	−1306.550 [−1403.690, −1209.41]	<0.00001
SAG	4	0	0.760	FEM	2.24 [1.78, 2.82]	<0.00001
LAG	4	87	<0.0001	REM	1.30 [0.53, 3.17]	0.57
Neonatal asphyxia	3	98	<0.00001	REM	5.08 [1.29, 20.06]	0.02
Neonatal hypoglycemia	3	41	0.180	FEM	2.86 [2.18, 3.75]	<0.00001
NRDS	2	94	<0.0001	REM	25.94 [5.42, 124.24]	<0.0001
Neonatal hyperbilirubinemia	2	0	0.780	FEM	5.41 [2.80, 10.45]	<0.00001
Neonatal death	3	0	0.400	FEM	5.33 [4.59, 6.19]	<0.00001

## Data Availability

Data appear in the submitted manuscript.

## References

[1] Retnakaran R., Shah B. R. (2016). Impact of twin gestation and fetal sex on maternal risk of diabetes during and after pregnancy. *Diabetes Care*.

[2] Weissman A., Drugan A. (2016). Glucose tolerance in singleton, twin and triplet pregnancies. *Journal of Perinatal Medicine*.

[3] Dillon J., Mitchell C. J., Ellett T., Siegel A., Denoble A. E., Dotters-Katz S. K. (2022). Pregnancy outcomes among women with class III obesity with pre-diabetic early hemoglobin A1C. *American Journal of Perinatology*.

[4] Buhling K., Henrich W., Starr E. (2003). Risk for gestational diabetes and hypertension for women with twin pregnancy compared to singleton pregnancy. *Archives of Gynecology and Obstetrics*.

[5] Jung Y. J., Kwon J. Y., Cho H. Y., Park Y. W., Kim Y. H. (2015). Comparison of the performance of screening test for gestational diabetes in singleton versus twin pregnancies. *Science*.

[6] Lai F. Y., Johnson J. A., Dover D., Kaul P. (2016). Outcomes of singleton and twin pregnancies complicated by pre-existing diabetes and gestational diabetes: a population-based study in Alberta, Canada, 2005–11. *Journal of Diabetes*.

[7] Rauh-Hain J. A., Rana S., Tamez H. (2009). Risk for developing gestational diabetes in women with twin pregnancies. *The Journal of Maternal-Fetal & Neonatal Medicine*.

[8] Akiba Y., Miyakoshi K., Ikenoue S. (2019). Glycemic and metabolic features in gestational diabetes: singleton versus twin pregnancies. *Endocrine Journal*.

[9] Morikawa M., Yamada T., Akaishi R. (2015). Prevalence of hyperglycaemia in singleton versus twin pregnancy. *Diabetes/Metabolism Research & Reviews*.

[10] Ashwal E., Berger H., Hiersch L. (2021). Gestational diabetes and fetal growth in twin compared with singleton pregnancies. *American Journal of Obstetrics and Gynecology*.

[11] González González N. L., González Dávila E., Goya M. (2014). Twin pregnancy among women with pregestational type 1 or type 2 diabetes mellitus. *International Journal of Gynaecology & Obstetrics the Official Organ of the International Federation of Gynaecology & Obstetrics*.

[12] Guillén-Sacoto M. A., Barquiel B., Hillman N., Burgos M. Á., Herranz L. (2018). Diabetes mellitus gestacional: control glucémico durante el embarazo y su relación con los resultados neonatales en embarazos gemelares y de feto único. *Endocrinología Diabetes Y Nutrición*.

[13] Hiersch L., Berger H., Okby R. (2018). Incidence and risk factors for gestational diabetes mellitus in twin versus singleton pregnancies. *Archives of Gynecology & Obstetrics*.

[14] Weiner E., Barber E., Feldstein O. (2018). The placental component and neonatal outcome in singleton vs. twin pregnancies complicated by gestational diabetes mellitus. *Placenta*.

[15] Borissov A. M., Trifonova B., Dakovska L., Michaylova E., Vukov M. (2021). Age, obesity, family history, previous gestational diabetes are major risk factors for hyperglycemia in pregnant Bulgarian women. *European Journal of Preventive Medicine*.

[16] Pirkola J., Pouta A., Bloigu A. (2010). Prepregnancy overweight and gestational diabetes as determinants of subsequent diabetes and hypertension after 20-year follow-up. *The Journal of Clinical Endocrinology and Metabolism*.

[17] Young C., Kuehl T. J., Sulak P. J., Allen S. R. (2000). Gestational diabetes screening in subsequent pregnancies of previously healthy patients. *American Journal of Obstetrics and Gynecology*.

[18] Xiao H. Y., Yu J., Liu Y. (2016). Gestational diabetes does not increase the risk of adverse perinatal outcome of twin pregnancy. *Chinese Journal of Perinatal Medicine*.

[19] Li Z. Y., Liu P. P., Zhu C. X., Chen H. T., Wang Z. L. (2016). Effect of gestational diabetes mellitus on perinatal outcome of double chorionic twins. *Journal of Sun Yat Sen University: Medical Science Edition*.

[20] Ooi S., Wong V. W. (2018). Twin pregnancy with gestational diabetes mellitus: a double whammy?. *Diabetes Care*.

[21] McGrath R. T., Hocking S. L., Scott E. S., Seeho S. K., Fulcher G. R., Glastras S. J. (2017). Outcomes of twin pregnancies complicated by gestational diabetes: a meta- analysis of observational studies. *Journal of Perinatology*.

[22] Sheehan A., Umstad M. P., Cole S., Cade T. J. (2019). Does gestational diabetes cause additional risk in twin pregnancy?. *Twin Research and Human Genetics*.

[23] Hiersch L., Berger H., Okby R. (2019). Gestational diabetes mellitus is associated with adverse outcomes in twin pregnancies. *American Journal of Obstetrics and Gynecology*.

